The article "Application Experience and Patient Feedback Analysis of 3D Printed AFO with Different Materials: A Random Crossover Study" was retracted in 2024. Reasons: signs of a paper mill; suspected computer-generated content; unreliable results or conclusions; concerns about the data.

# Application Experience and Patient Feedback Analysis of 3D Printed AFO with Different Materials: A Random Crossover Study

**DOI:** 10.1155/2021/8493505

**Published:** 2021-06-12

**Authors:** Xianzhong Meng, Min Ren, Yan Zhuang, Yu Qu, Linling Jiang, Zhenjing Li

**Affiliations:** Department of Rehabilitation, Pudong New Area People's Hospital, China

## Abstract

**Purpose:**

This study is aimed at analyzing the application experience and feedback of the patients with poststroke ankle dorsiflexion disorders for 3D printed AFO with three different materials.

**Methods:**

15 patients were randomly divided into three groups; 3D printed AFO with 3 different materials (PA2200, Somos NeXt, and PA12) was used to each group, according to the crossover study design, in order to ask the three groups of patients to use three different materials of 3D printed AFO. Assessment was taken by the end of each test round. Through statistical processing, the patient feedback data of the three groups of materials of 3D printed AFO were obtained.

**Results:**

In the material comfort assessment of the AFO, Somos NeXt was compared with PA2200, and the *p* value was <0.05; in the item of surface smoothness of the AFO, Somos NeXt was compared with PA2200, and the *p* value was <0.01; at the same time, PA12 was compared with PA2200, and the *p* value was <0.05.

**Conclusion:**

The 3 different materials of 3D printing AFO bring different experience, and we also have sufficient reason to believe that there will be differences in the auxiliary effect of this on patients, which leads the patient's selection too. The material Somos NeXt is much popular and has certain clinical advantages.

## 1. Introduction

Three-dimensional printing (3D) is one of additive manufacturing technologies, which appeared in the 1980s. It establishes the 3D data of the target model by means of CT, MRI, CAD, or 3D scanning, processes it into a 3D digital model file by reverse engineering modeling software, then transmits it to a suitable printer, and finally selects suitable materials to print the target model layer by layer. Because 3D printing technology has the advantages of personalized customization, the ability to manufacture complex and fine structures, high material utilization, and short manufacturing cycle has been widely used in the medical field, such as the application of ankle foot orthosis (AFO) in rehabilitation medicine. Poststroke patients are often accompanied by paralysis of the lower limbs, foot drop, and varus [1]. For these patients with ankle dorsiflexion disorders, the configuration of AFO can effectively improve hemiplegic gait and improve walking function. However, there are some defects in traditional orthoses, such as the inability to achieve personalized design for plaster or splint fixation, and may cause serious skin infections, limb stiffness, pressure sores, and other complications; low-temperature thermoplastic plates need to be adjusted repeatedly when manufacturing orthoses, which has the risk of scalding patients; the manufacturing process of high-temperature plastic orthosis is cumbersome, the efficiency is low, and the appearance is unsightly [2]. 3D printing technology completes the construction of the whole entity through layered processing and superposition molding, which can achieve design freedom and can be optimized according to personal biomechanical requirements to provide patients with better orthopedic functions and better appearance design [3]. 3D printing AFO may improve patient satisfaction, wearing compliance, and the quality of life of patients [4].

The commonly used materials for 3D printers include plastics, metals, resins, nylon, hydrogels, ceramics, and composite. Currently, the most commonly used technologies include stereo lithography appearance (SLA), fused deposition modeling (FDM), selective laser sintering/melting (SLS/SLM), laminated object manufacturing (LOM), and three-dimensional jet printing (3DP) [5]. This study is aimed at comparing the actual printing effects of the three commonly used printing materials for orthotics and exploring their application experience and feedback in patients with poststroke ankle dorsiflexion disorders [6].

Crossover design is normally used as another important study design for clinic trial when the study needs the patients to use two or more interventions, allowing the patient to compare themselves. Its advantage is that the same patient receives two or more interventions successively and obtains two or more results; this type of design can reduce the number of samples, and it has better ethics and economics [7]. However, due to the washout period and sequential clinical intervention steps, crossover study design also has disadvantages: (a) it is only suitable for symptomatic treatment of chronic recurrent diseases; (b) observation time is prolonged, and patients are likely to be lost to follow up, withdraw, and decline compliance; (c) research on diseases that are not suitable for acute onset and short course of disease. It is precisely because of the characteristics of crossover design that this type of design is suitable for this study [8].

## 2. Clinical Data

### 2.1. Research Object and Grouping

Patients with poststroke ankle dorsiflexion disorders in the Rehabilitation Department of the Shanghai Pudong New Area People's Hospital from July 1, 2020, to December 31, 2020. Finally, according to the inclusion and exclusion criteria, a total of 15 subjects were determined and randomly divided into three groups: group A, group B, and group C.

### 2.2. Diagnostic Criteria

The diagnostic criteria of stroke were formulated with reference to the Chinese Guidelines for Diagnosis of various cerebrovascular diseases.

### 2.3. Inclusion Criteria

The inclusion criteria of this study were as follows: (1) a minimum of 3-month poststroke with hemiparesis; (2) an ability to walk safely with the use of an AFO; (3) participation is voluntary, and informed consent has been signed.

### 2.4. Exclusion Criteria

The exclusion criteria of this study were as follows: (1) patients with severe pain or musculoskeletal issues and (2) patients with cognitive issues [9].

## 3. Intervention and Crossover Design

### 3.1. Data Acquisition and Preparation before Brace 3D Printing

Artec and 3D scanner (EinScan-Pro, Shining 3D scanner company) were used to scan the legs, ankles, and feet of paralyzed limbs. Sitting or lying position was required. After scanning, the initial AFO 3D model image can be obtained. Then, the software Geomagic Studio was used to modify, and surface treatment of the AFO model (STL file type) designed a reasonable AFO shape; the key processing procedures include the following: according to the design requirements, deleted the extra patch; used tools of “Remove Feature,” “Fill Single Hole,” “Fill All,” and other tools to repair the broken hole; smoothed boundary lines and set thickness value.

### 3.2. Brace 3D Printing with Different Materials

After the design was completed, the AFO model was output in STL file format, and the required AFO was printed by a 3D printer. This study involved 3 different materials: PA2200 [10], Somos NeXt [11], and PA12 [12]. The material PA2200 is characterized by high strength, light weight, and toughness, and the printing method is SLS [10]. The material Somos NeXt is white, with high strength and toughness and good precision and appearance, and the printing method is SLA [11]. The material PA12 has extremely low moisture absorption, excellent mechanical strength, and good wear resistance and corrosion resistance, and the printing method is MJF [12].

### 3.3. Crossover Design

Random grouping was carried out according to the patient's medical record number. The 15 patients' medical record numbers were arranged from small to large, so that every five persons were divided into a group. Three groups were set, group A, group B, and group C. Each group had 5 patients. The patients were all informed and signed an informed consent, respectively [7].

During the experiment, the patients would not know the specific plan of the material used in the brace, and they only be notified that a new brace would be replaced after the washout period, in order to set up blind barriers [7].

From the beginning, we set group A to use 3D printing AFO with material 1, group B to use 3D printing AFO with material 2, and group C to use 3D printing AFO with material 3. After wearing for one week, all the patients have 2 days to take a pause for rest and also for the wash-out period. Next, group B took material 1, and group C took material 2, while group A took material 3, wearing one week and two-day wash-out period. In the last round, group C took material 1, group A took material 2, and group B took material 3, wearing one week. The assessment points would be on the last day of each round [7]. See Figure 1.

## 4. Evaluation

(1) *Evaluation Items*. The study sets 7 assessment items as shown below:
  - Material comfort assessment of the AFO
  - Weight feeling of the AFO
  - Surface smoothness of the AFO
  - Difficulty in wearing
  - Convenience of cleaning
  - Skin lesion
  - The occurrence of adverse events

We set up score sheets for each assessment item above, and the NRS system concept was used. The 100 was set as prefect, while the 0 was set as the worst. See Figure 2.

(2) *Evaluation Points*. The assessment points would be on the last day of each wearing round. It meant the day 7, day 16, and day 25.
(3) The evaluation was made by an independent researcher; she collected the data with self-sufficient and contacted with the study participants

## 5. Statistical Methods

Data of material comfort, weight, surface smoothness, difficulty in wearing, convenience of cleaning, and skin lesion were collected in on MS Excel file, and material classification as a parameter was used to integrate three parts of data. With the IBM SPSS 22.0 Statistics Software, one-way ANOVA LSD and T3 were used to detect the difference among the three parts, in order to make decision whether the three parts of data were able to merge. After that, three types of different materials of 3D printing AFO feedback data were received. Based on these feedback data of three materials, each material data had 7 parameters, which were also the 7 comparison items mentioned above. One-way ANOVA was taken again to make a statistical analysis.

## 6. Results

1. The possibility of data merge

Taking the material as the parameter, groups A, B, and C provided three parts of the data, and the comparison results showed that there was no significant difference among the three parts. It indicated that the order of wearing had no correlation with the brace data of different materials.

(2) After data merge, three types of different materials of 3D printing AFO feedback data were received. The comparison results are indicated in the material comfort assessment of the AFO; Somos NeXt was compared with PA2200, and the *p* value <0.05 means there is a significant difference; in the item of surface smoothness of the AFO, Somos NeXt was compared with PA2200, and the *p* value <0.01 means there is a great significant difference, and at the same time, PA12 was compared with PA2200, and the *p* value <0.05 means a significant difference. See Figures 3 and 4 and Table 1

## 7. Discussion

AFO can effectively improve the kinematics and dynamics parameters of the ankle and knee joints and is mainly used for walking and correcting deformities of drooping feet and clubfoot. The preparation of traditional AFO relies on handwork, which requires a high level of skill and a lot of meticulous work by the maker; however, with 3D printing technology, we only need to enter the design parameters once, which can be used for life, which greatly facilitates the replacement and adjustment of subsequent orthotics. AFO printed by 3D has high design flexibility and strong personalized customization ability, which can put on “beautiful shoes” for patients and improve their self-confidence. Cha et al. [13] designed a 3D printed AFO for a 68-year-old female foot drop patient and compared the use effect with the traditional AFO, and the results show that 3D printed AFO can make the patient's left and right foot posture more symmetrical when walking, that is, walking is more natural and stable; moreover, 3D printed AFO has a better effect on preventing foot drop and is easier to wear than traditional AFO.

The printing method of 3D printing and the material properties of the printing materials are important factors that affect the printing effect. In recent years, some studies have adopted different printing materials, carried out some mechanical tests including accuracy and bending strength, and conducted a few clinical studies. Mavroidis et al. [6] established the AFO model by scanning ankle and foot with 3D scanner and printed AFOs of two different materials. One AFO which was printed of Accura 40 resin was hard, and the other which was printed of DSM Somos 9120 was soft. Both of the AFOs have high precision and the same clinical effects compared with traditional AFO products [3].

Crossover design's advantage application to that the same patient can receive different interventions at different stages, and the washout period between the two interventions effectively blocks the delayed effects of the interventions. In this study, the AFO brace function is the same, but made from 3 different materials. The brace itself does not have a long-term delayed effect on patients; therefore, this study does not require a long washout period [2, 8]. The same patient tries 3 different materials of AFO braces, and each patient's comparative data comes from herself/himself, which objectively guarantees the consistency of subjective feelings, which plays a vital role in the stability and accuracy of experimental data. Randomly dividing into three groups, to a certain extent, avoided the impact of the intervention sequence of the three different materials of 3D printed braces on the subjective feelings of the patients and increased the comparability of the data.

It can be learned from this study that the actual printing effects of the three materials are different. In this experiment, we used 3 printing methods to print 3 different materials; Somos NeXt used SLA printing, PA2200 used SLS printing, and PA12 used MJF printing. All AFOs have high accuracy, which matches the ankle and foot of patients. This result is consistent with the expectations, reflecting the advantages of 3D printing technology and meeting the technical parameters of the three materials. From the view of material comfort and surface smoothness, PA2200 gets the lowest score, while the Somos NeXt gets the highest; this is certainly related to the printing method, but it also reveals the disadvantages of this material. Participants' feedback also shows Somos NeXt is the easiest for wearing and cleaning. No skin lesion and adverse events happened [10–12].

In summary, the 3 different materials of 3D printing AFO bring different experience, and we also have sufficient reason to believe that there will be differences in the auxiliary effect of this on patients, which leads the patient's selection too. The material Somos NeXt is much popular and has certain clinical advantages.

## Figures and Tables

**Figure 1:** Crossover study design.

**Figure 2:** NRS system concept.

**Figure 3:** Comparison histogram among different materials.

**Figure 4:** Comparison radar map among different materials.

**Table 1:** Three different material comparison data.

	PA2200 mean (SD)	Somos NeXt mean (SD)	PA12 mean (SD)
Material comfort assessment of the AFO	42.73 (30.52)	75.31 (26.88)^∗^	59.22 (36.01)
Weight feeling of the AFO	57.65 (10.63)	59.06 (16.91)	57.13 (20.82)
Surface smoothness of the AFO	37.40 (9.05)	85.26 (17.80)^∗∗^	60.27 (28.11)^∗^
Difficulty in wearing	70.18 (19.66)	79.06 (27.05)	77.91 (30.01)
Convenience of cleaning	80.69 (6.02)	85.07 (10.22)	83.00 (11.74)
Skin lesion	None	None	None
Adverse events	None	None	None

^∗^Compared with PA2200, *p* < 0.05; ^∗∗^compared with PA2200, *p* < 0.01.

## Data Availability

The study data used to support the findings are kept by the project team data center of Pudong New Area People's Hospital, and requests for data will be considered by the data center.

## References

[1] Liaw C. Y., Guvendiren M. (2017). Current and emerging applications of 3D printing in medicine. *Biofabrication*.

[2] Fan D., Li Y., Wang X. (2020). Progressive 3D printing technology and its application in medical materials. *Frontiers in Pharmacology*.

[3] Tack P., Victor J., Gemmel P., Annemans L. (2016). 3D-printing techniques in a medical setting: a systematic literature review. *Biomedical Engineering Online*.

[4] Herbert N., Simpson D., Spence W. D., Ion W. (2005). A preliminary investigation into the development of 3-D printing of prosthetic sockets. *Journal of Rehabilitation Research and Development*.

[5] Katsuhira J., Yamamoto S., Machida N. (2018). Immediate synergistic effect of a trunk orthosis with joints providing resistive force and an ankle-foot orthosis on hemiplegic gait. *Clinical Interventions in Aging*.

[6] Mavroidis C., Ranky R. G., Sivak M. L. (2011). Patient specific ankle-foot orthoses using rapid prototyping. *Journal of Neuroengineering and Rehabilitation*.

[7] Nolan S. J., Hambleton I., Dwan K. (2016). The use and reporting of the cross-over study design in clinical trials and systematic reviews: a systematic assessment. *PLoS One*.

[8] Tyson S. F., Sadeghi-Demneh E., Nester C. J. (2013). A systematic review and meta-analysis of the effect of an ankle-foot orthosis on gait biomechanics after stroke. *Clinical Rehabilitation*.

[9] Chinese Society of Neurology, Chinese Society of Neurosurgery (1996). Diagnostic essentials of various cerebrovascular diseases. *Chinese Journal of Neurology*.

[10] EOS Inc.: products-PA2200. https://eos.materialdatacenter.com/eo/en/PA2200material.pdf.

[11] DSM Inc.: products-Somos NeXt. https://www.dsw.com/solutions/additivemanufacturing/en_US/products/for-stereolithography/somos-next.htm.

[12] HP Inc.:Products-PA12. https://www8.hp.com/us/en/printers/3d-printers/materials.html.

[13] Cha Y. H., Lee K. H., Ryu H. J. (2017). Ankle-foot orthosis made by 3D printing technique and automated design software. *Applied Bionics and Biomechanics*.

